# Study on Huangqi Bazhen Decoction on Relieving Chemotherapy Intestinal Mucositis in Capecitabine Gavage Mice

This article has been retracted.

**DOI:** 10.1155/2022/3826080

**Published:** 2022-09-28

**Authors:** Tieyi Shi, Baozhong Chen, Cheng Liu, Ker Lu

**Affiliations:** College of Basic Medicine, Heilongjiang University of Chinese Medicine, Harbin 150040, China

## Abstract

In order to provide evidence for clinical application, the therapeutic effect and mechanism of Huangqi Bazhen decoction on chemotherapeutic intestinal mucositis induced by capecitabine in mice are investigated. In this paper, the mice are divided into different groups and given capecitabine intragastric administration or treatment drugs. Morphological features of intestinal injury, including villus height shortening, crypt destruction, and apoptosis, are reversed. The experimental results show that Huangqi Bazhen decoction can significantly reduce weight loss and diarrhea during capecitabine treatment. It is also found that GSH-Px and T-SOD can be improved while MDA, IL-1*β*, and TNF-*α* are reduced significantly.

## 1. Introduction

As a pyrimidine chemotherapeutic agent, capecitabine is commonly used to treat colon and breast cancer. It is relatively non-cytotoxic in vitro and can inhibit tumor growth by inhibiting cell division and interfering with protein synthesis. However, it may cause adverse reactions such as vomiting and diarrhea [1]. Clinical data show that the incidence rate of severe diarrhea is 20% approximately, and it is easy to cause patient dose dependence [2, 3]. The clinical symptoms of chemotherapy-induced intestinal mucositis (CIM) are nausea, vomiting, diarrhea, and abdominal pain. The pathological features are villus destruction, crypt damage, and inflammatory cell infiltration [4]. Chemotherapy-induced intestinal mucositis brings great pain to patients, reduces chemotherapy compliance, and hinders clinical work. Generally, patients can relieve symptoms by reducing the dose of chemotherapy, but it will seriously affect the progress of tumor treatment [5]. Traditional Chinese medicine (TCM) plays an important role in the treatment and recovery of gastroenteritis with its unique diagnosis, treatment methods, and concepts [6]. It should be noted that cancer patients suffer from a variety of diseases and chronic physical failure. In recent years, TCM clinical workers have gradually realized the importance of prevention and treatment based on tonic, and prevention has gradually become an effective means to alleviate the side effects of chemotherapy [7]. Clinically, Huangqi Bazhen decoction is often used in combination with chemotherapy drugs to reduce adverse reactions. In addition, TCM can supplement stomach Qi in time when the disease is not invaded and play a role in resisting external pathogens [8].

In order to provide evidence for clinical application, the therapeutic effect and mechanism of Huangqi Bazhen decoction on chemotherapeutic intestinal mucositis induced by capecitabine in mice are investigated. These results indicate that the mechanism of Huangqi Bazhen decoction in treating chemotherapeutic intestinal mucositis may be through inhibition of apoptosis signal transduction pathway and reduction of apoptosis.

The rest of the paper is organized as follows.  Section 2 discusses related studies.  Section 3 introduces the materials and proposed method. The results and analysis are discussed in Section 4.  Section 5 serves as a conclusion, providing the summary and future directions of research.

## 2. Related Work

The gastrointestinal mucosa is easily damaged by chemotherapy. After the gastrointestinal mucosa is damaged, there will be inflammation of the gastrointestinal mucosa, which will lead to a series of gastrointestinal reactions such as nausea, vomiting, diarrhea, and abdominal distension. The pathological features of CIM include villus destruction, crypt damage, and inflammatory cell infiltration [9, 10]. Moreover, further damage to the intestinal mucosa also increases permeability. Furthermore, it damages the immune barrier, causes bacterial imbalance, leads to poor blood, and aggravates systemic inflammation. Inflammatory changes of rectal mucosa will also increase the possibility of gastrointestinal ulcer, bleeding, and perforation, which has a certain risk.

IL-1*β* is an inflammatory factor formed by caspase-1-cleaved IL-1*β* precursors activated by NLRP3. In this way, the body responds to microbial infection and cell damage. At the same time, activated caspase-1 activates gasdermin D to perforate the cell membrane, releasing inflammatory factors such as IL-1*β* and causing severe inflammatory reaction [11]. This lack of control of inflammatory mediators can cause chronic inflammation to persist and cause mucositis in the digestive tract. Tumor necrosis factor (TNF) is a multifunctional proinflammatory cytokine and immunomodulator that functions by activating two different receptors, TNFR1 and TNFR2. TNF-*α* activates classical and non-classical NF-*κ*B pathways and JNK/MAP kinase signaling and drives inflammation, cell proliferation, and cell survival [12] by binding to receptors. On the other hand, depending on the cellular environment, TNFR1 also activates apoptotic signaling pathways leading to cell death [13].

Oxidative stress is closely related to inflammatory responses. When stimulated, the phagocyte breathes out, consumes oxygen, and releases superoxide anion, hydrogen peroxide, and other substances to directly injure endothelial cells, erythrocytes, fibroblasts, and platelets. ROS also induces apoptosis. Radiation, inflammation, macrophage activation, and other processes will produce a large number of ROS. These ROS are mainly generated in mitochondria, resulting in lipid peroxidation, damage to DNAs, activation of NF-*κ*B, and activation of apoptosis signals. They can also stimulate TNFR to activate NADPH oxidase. Oxygen free radicals increase rapidly. Mitochondria are extremely sensitive to reactive oxygen. After accumulation of excessive ROS in cells, mitochondria membrane permeability changes, membrane potential decreases, and cytochrome C is released, resulting in apoptosis [14].

Capecitabine acts as an antitumor agent by interfering with the cell cycle while damaging normal cells [15]. In jejunum tissue, goblet cells can secrete mucin, which can lubricate the intestine and prevent toxic substances from invading. Chemotherapy drugs are excreted into jejunum tissue with bile after liver metabolism, and a large number of intestinal crypts are damaged, so the differentiation of various intestinal cells is blocked. Among them, goblet cell injury leads to reduction of intestinal protective protein secretion, and intestinal injury will be further aggravated. Related experiments showed that pathological section of 5-FU model mice showed increased expression of inflammatory factor in jejunum tissue, increased apoptosis of jejunum tissue under electron microscope, and increased expression of caspase-3 protein in jejunum tissue, indicating that intestinal mucositis caused by pyrimidines is related to apoptosis of jejunum cell [16].

## 3. Materials and Proposed Method

### 3.1. Materials

#### 3.1.1. Instrument

The instruments are as follows: 2135 microtome (Leica Microsystems, Trading Co. Ltd.), Moticam 3000 microphotographic system (McAudi Industrial Group Co. Ltd.), electric thermostat (Shanghai Yi Heng Science & Technology Co. Ltd.), DNM-9602 microplate reader (Beijing Plang Co. Ltd.), Type DNX-96 isher (Beijing Plang Co., Ltd.), electronic balance (PL 602-L) (Meterler Toledo Instrument Co. Ltd.) and TGL-16G table centrifuge (Shanghai Anting Scientific Instrument Factory).

#### 3.1.2. Drugs and Reagents

The drugs and reagents include IL-1*β* Mouse ELISA Kit and TNF-*α* Mouse ELISA Kit (Beijing Chenglin Biotechnology Company, China), Rabbit anti-caspase-3 polyclonal antibody and Rabbit anti-caspase-8 polyclonal antibody (Beijing Boorson Biotechnology Company, China), PV two-step method and DAB developer (Beijing Zhongshan Golden Bridge Biotechnology Company, China), TUNEL Apoptosis Detection Kit (Roche Pharmaceutical Company), SOD determination kit, MDA determination kit and GSH-PX determination kit (Nanjing Jiancheng Bioengineering Institute, China), BCA protein quantitative kit (Shanghai Biyuntian Biotechnology Company, China), capecitabine tablets (trade name: Zhuolun, manufactured by Qilu Pharmaceutical Company, specification: 0.5 g/tablets, batch number: Sinopharm No. H20133361), montmorillonite powder (trade name: Smecta, manufactured by Bofu-Ipson Pharmaceutical Company, specification: 3 g/bags, batch number: Sinopharm H20000690).

#### 3.1.3. Experimental Animals

SPF ICR mice (male, weight 18–22 g, and animal license number: SYXK (black) 2018-003) were provided by Experimental Animal Center of Heilongjiang University of Traditional Chinese Medicine. The mice are fed and managed in the laboratory, the room temperature is 24 ± 3°C, and the relative humidity is controlled at 50∼60%.

### 3.2. Proposed Method

#### 3.2.1. Preparation of Chinese Medicine

Radix Angelicae Sinensis, Rhizoma Chuanxiong, Radix Rehmanniae Preparata, Radix Paeoniae Alba, Radix Codonopsis, Radix Glycyrrhizae Preparata, Poria cocos, Rhizoma Atractylodis Macrocephalae, and Radix Astragali were purchased from the Chinese Medicine Department of the First Affiliated Hospital of Heilongjiang University of Chinese Medicine. Firstly, mix the medicines and add eight times the amount of distilled water. Then, after boiling for 40 minutes, pour out the liquid. Subsequently, add six times the amount of distilled water and decoct for 30 min. Mix and filter the medicinal liquid twice and finally concentrate the dose of Chinese medicine to 5 g/mL with 4°C. Bath to 37°C before use.

#### 3.2.2. Grouping, Modeling, and Administration of Experimental Animals

40 male ICR mice are fed adaptively for 3 days. The mice are divided into control group, capecitabine group, montmorillonite powder group, and Huangqi Bazhen decoction (HQBZD) treatment group. In the control group, the normal saline is intragastrically administered twice according to 0.1 ml/10 g, with an interval of half an hour. The capecitabine group is given capecitabine solution by gavage at 200 mg/kg and normal saline by gavage at 0.1 ml/10 g after half an hour. The montmorillonite powder group is perfused with capecitabine and the montmorillonite powder (1.2 g/kg). HQBZD group is given capecitabine liquid and HQBZD (50 g/kg) by gavage.

#### 3.2.3. Sampling of Experimental Animals

On the 12th day, one hour after oral gavage, blood is taken from the eyes, 3000 r/min is centrifuged for 15 min, and the supernatant is taken. After the mice are sacrificed, the abdominal cavity is opened, and 2 cm of intact jejunal tissue is taken at 15 cm of the lower part of the pylorus, fixed in 4% paraformaldehyde, and then embedded in paraffin.

#### 3.2.4. Weight Change and Diarrhea Index of Mice

The mice will be weighed on days 1, 4, 8, and 12. Diarrhea degree is scored on the 8th, 10th, and 12th day, and diarrhea index is calculated according to the Kurita method. Normal stool or no score is 0. Mild diarrhea, mild stool wet soft score is 1. Moderate diarrhea, no stool formation, mild perianal staining 2 points. Severe diarrhea, watery stool, severe perianal staining 3 points. Diarrhea index can be calculated by the ratio of the sum of diarrhea scores per mouse in group to the number of mice in group.

#### 3.2.5. Detection of Apoptosis by TUNEL Staining

Take 100 *μ*L marker solution from reagent 2 as negative control. All of the liquid in reagent 1 is added to the remaining labeling solution in reagent 2 to form a reaction mixture. Paraffin slices are routinely dewaxed to water. Add pepsin K (20 *μ*g/ml in 10 mM Tris/HCL, pH 7.4–8.0) dropwise, incubate at room temperature for 30 min, and rinse twice. Dry the water around the sample, add 50 *μ*L of TUNEL reaction mixture dropwise, incubate for 60 min in a wet box with 37°C, and rinse three times with PBS. Dry the water around the sample, incubate for 30 min in the wet box with 37°C, and rinse three times.

#### 3.2.6. Immunohistochemical Detection of Caspase-3 and Caspase-8 Protein Expression in Tissues

In this paper, the average integrated optical density is used to express the relative expression of proteins. Each group randomly analyzes 6 high-power fields to represent the average relative expression of photos. The staining result showed that the nuclei are blue and the positive ones are yellow or yellowish brown.

### 3.3. Statistical Analysis

SPSS 20.0 statistical analysis software package is used for processing, $\bar{x}\pm s$ is used for description of indexes, *t* test is used for comparison of indexes between two groups, and single-factor analysis of variance is used for comparison of indexes between multiple groups. When *P* < 0.05, the difference is statistically significant, and when *P* < 0.01, the difference is statistically significant.

## 4. Results and Analysis

### 4.1. Mouse Body Weight Change and Diarrhea Index

The body weight of mice at days 1, 4, 8, and 12 is analyzed. On the 4th day, the body weight of each group increased to different degrees, and the body weight of HQBZD group is higher than that of capecitabine group (*P* < 0.05). On the 8th day, the number of HQBZD group is significantly higher than that of capecitabine group (*P* < 0.01). On the 12th day, the weight of HQBZD group and montmorillonite powder is significantly higher than that of capecitabine group (*P* < 0.01).

In terms of diarrhea index, on the 8th day, the diarrhea degree of each treatment group is not significantly changed compared with capecitabine group (*P* > 0.05); on the 10th day, the diarrhea degree of HQBZD group is improved compared with capecitabine group (*P* < 0.05); on the 12th day, the diarrhea degree of montmorillonite powder group and HQBZD group is significantly improved compared with capecitabine group (*P* < 0.01), as shown in Tables 1 and 2.

### 4.2. Histopathological Observation of Jejunum and Intestinal Villus Height and Crypt Depth

In the capecitabine group, the villi of intestine became short, the crypt depth became shallow, and inflammatory cells infiltrated. The damage degree of jejunum tissue in the montmorillonite powder group is lighter than that of the capecitabine group, the intestinal villus is complete, the crypt depth is deep, and the inflammatory cell infiltration is reduced. The damage degree of jejunum tissue is reduced in HQBZD groups, the villus of intestine is intact, the crypt is deep, and the inflammatory cell infiltration is reduced.

The villus height and crypt depth of jejunum in the capecitabine group are significantly lower than those in the control group (*P* < 0.01). The villi height and crypt depth of jejunum tissue in HQBZD group are significantly higher than those in the capecitabine group (*P* < 0.01). It indicates that Huangqi Bazhen decoction can reduce the villi height and crypt depth of jejunum tissue in mice induced by capecitabine, as shown in Figure 1 and Table 3.

### 4.3. Determination of IL-1*β*, TNF-*α*, GSH-PX, MDA, and T-SOD in Serum of Mice

The contents of IL-1*β*, TNF-*α*, and MDA in the serum of capecitabine group are significantly higher than those of the control group (*P* < 0.01). The content of IL-1*β*, TNF-*α*, and MDA in montmorillonite powder group is lower than that in the capecitabine group, but there is no difference (*P* > 0.05). The contents of IL-1*β*, TNF-*α*, and MDA in the HQBZD group are significantly lower than those in the capecitabine group (*P* < 0.01). The contents of GSH-PX and T-SOD in the capecitabine group are significantly lower than those in the control group (*P* < 0.01). Montmorillonite powder group had no statistical significance compared with capecitabine group (*P* > 0.05). The contents of GSH-PX and T-SOD in the HQBZD group are significantly higher than those in the capecitabine group (*P* < 0.01), which indicated that Huangqi Bazhen decoction could significantly reduce the inflammatory reaction, relieve the increase of oxidative stress level in mice induced by capecitabine, and enhance the antioxidant capacity of mice, as shown in Table 4.

### 4.4. Apoptosis and Expression of Caspase-3 and Caspase-8 Protein in Jejunum of Mice

Compared with the control group, apoptosis and caspase-3 and caspase-8 expression increased in the capecitabine group (*P* < 0.01). Compared with the capecitabine group, apoptosis and caspase-3 and caspase-8 expression in the montmorillonite powder group decreased significantly (*P* < 0.01). The apoptosis and the expression of caspase-3 and caspase-8 in the HQBZD group are significantly lower than those in the capecitabine group (*P* < 0.01), as shown in Table 5.  Figure 2 shows the apoptosis and expression of caspase-3 protein in jejunum of mice.  Figure 3 shows the apoptosis and expression of caspase-8 protein in jejunum of mice.

## 5. Conclusions

It can cause damage of jejunal tissue structure and inflammatory cell infiltration, significantly increase expression of IL-1*β* and TNF-*α* inflammatory factor in serum, and significantly increase oxidative stress level of GSH-PX, T-SOD, and MDA. Huangqi Bazhen decoction can reduce inflammatory cell infiltration in jejunal tissue, protect intestinal structural integrity, and have therapeutic effect on chemotherapeutic intestinal mucositis. It is suggested that Huangqi Bazhen decoction could reduce inflammatory reaction and oxidative stress level and reduce damage of inflammatory factor and active oxygen to jejunal tissue. The results of TUNEL and immunohistochemistry show that Huangqi Bazhen decoction could reduce apoptosis and the expression of caspase-3 and caspase-8 in jejunum tissue. The observations indicate that the mechanism of Huangqi Bazhen decoction in treating chemotherapeutic intestinal mucositis may be through inhibition of apoptosis signal transduction pathway and reduction of apoptosis.

## Figures and Tables

**Figure 1:** Histopathological observation of jejunum and intestinal villus height and crypt depth: (a) control group; (b) capecitabine group; (c) montmorillonite powder group; (d) HQBZD group.

**Figure 2:** Apoptosis and expression of caspase-3 protein in jejunum of mice: (a) control group; (b) capecitabine group; (c) montmorillonite powder group; (d) HQBZD group.

**Figure 3:** Apoptosis and expression of caspase-8 protein in jejunum of mice: (a) control group; (b) capecitabine group; (c) montmorillonite powder group; (d) HQBZD group.

**Table 1:** Effect of Huangqi Bazhen decoction on weight of mice induced by capecitabine ($\bar{x}\pm s$, *n* = 10).

Group	Mean body weight change/g			
	Day 1	Day 4	Day 8	Day 12
Control	23.30 ± 0.92	26.90 ± 0.88^*∗∗*^	29.41 ± 1.30^*∗∗*^	30.27 ± 0.96^*∗∗*^
Capecitabine	23.87 ± 0.88	24.13 ± 0.84	22.07 ± 0.74	20.55 ± 0.73
Montmorillonite powder	23.35 ± 1.22	24.03 ± 1.21	22.90 ± 1.15	21.97 ± 1.12^*∗∗*^
HQBZD	23.25 ± 0.83	24.90 ± 0.48^*∗*^	25.07 ± 1.05^*∗∗*^	24.43 ± 1.34^*∗∗*^

^∗∗^ *P*<0.01, ^∗^*P*<0.05.

**Table 2:** Effect of Huangqi Bazhen decoction on diarrhea induced by capecitabine in mice ($\bar{x}\pm s$, *n* = 10).

Group	Day 8	Day 10	Day 12
Control	0	0	0
Capecitabine	0.8 ± 0.6	1.6 ± 0.8	2.4 ± 0.49
Montmorillonite powder	0.3 ± 0.46	1.1 ± 0.7	1.3 ± 0.46^*∗∗*^
HQBZD	0.3 ± 0.46	0.7 ± 0.64^*∗*^	1.2 ± 0.6^*∗∗*^

**Table 3:** Effects of Huangqi Bazhen decoction on villus height and crypt depth in jejunum of mice ($\bar{x}\pm s$, *n* = 10).

Group	Height of villus (Um)	Crypt depth (Um)
Control	288.75 ± 24.68^*∗∗*^	166.17 ± 11.41^*∗∗*^
Capecitabine	200.42 ± 13.90	91.85 ± 7.53
Montmorillonite powder	252.58 ± 14.86^*∗∗*^	131.59 ± 9.05^*∗∗*^
HQBZD	272.05 ± 18.38^*∗∗*^	140.41 ± 13.74^*∗∗*^

**Table 4:** Effects of Huangqi Bazhen decoction on IL-1*β*, TNF-*α*, GSH-PX, T-SOD, and MDA in serum of mice ($\bar{x}\pm s$, *n* = 10).

Group	IL-1*β* (Ng/L)	TNF-*α* (Ng/L)	GSH-PX (Mmol/L)	T-SOD (U/ml)	MDA (Mmol/L)
Control	47.18 ± 5.97^*∗∗*^	18.25 ± 2.25^*∗∗*^	50.02 ± 4.35^*∗∗*^	202.32 ± 9.08^*∗∗*^	5.54 ± 0.99^*∗∗*^
Capecitabine	77.66 ± 5.52	55.22 ± 4.84	22.01 ± 2.70	86.02 ± 6.70	10.19 ± 1.24
Montmorillonite powder	72.54 ± 5.2	50.18 ± 3.32	25.11 ± 3.38	96.23 ± 8.6	8.97 ± 0.73
HQBZD	50.75 ± 4.69^*∗∗*^	25.66 ± 3.34^*∗∗*^	46.32 ± 5.14^*∗∗*^	177.14 ± 8.33^*∗∗*^	6.99 ± 0.41^*∗∗*^

**Table 5:** Effects of Huangqi Bazhen decoction on apoptosis and expression of caspase-3 and caspase-8 protein in jejunum of mice ($\bar{x}\pm s$, *n* = 10).

Group	TUNEL (number)	Caspase-3 (IOD/area)	Caspase-8 (IOD/area)
Control	11.83 ± 2.11^*∗∗*^	29.73 ± 3.21^*∗∗*^	43.32 ± 5.44^*∗∗*^
Capecitabine	40.83 ± 3.48	79.485 ± 8.06	90.12 ± 6.64
Montmorillonite powder	25.33 ± 1.97^*∗∗*^	49.46 ± 5.51^*∗∗*^	56.93 ± 6.66^*∗∗*^
HQBZD	22.17 ± 2.79^*∗∗*^	46.06 ± 4.67^*∗∗*^	54.37 ± 4.59^*∗∗*^

## Data Availability

The simulation experiment data used to support the findings of this study are available from the corresponding author upon request.
